The article "Impact Sound Insulation Performance Testing of Nano-Inorganic Composite Floor Slabs for Green Buildings" was retracted in 2023. Reasons: signs of a paper mill; suspected computer-generated content; unreliable results or conclusions; concerns about the data.

# Impact Sound Insulation Performance Testing of Nano-Inorganic Composite Floor Slabs for Green Buildings

**DOI:** 10.1155/2022/5642361

**Published:** 2022-08-24

**Authors:** Weibing Luo, Yigang Yang, Hongyan Zhou

**Affiliations:** College of Architectural Engineering, Jiangxi Vocational College of Finance and Economics, Jiujiang, Jiangxi 332000, China

## Abstract

To explore the detection of impact sound insulation performance of nano-inorganic composite floor slabs for green buildings, for 4 types of floor slab practices in a certain area, we carry out the detection of the sound insulation performance of the floor impact sound and analyze and summarize the test results. Finally, several common technical measures to effectively improve the sound insulation performance of floor impact sound are summarized. Experimental results show that with floor slabs using nano-inorganic composite material FBP, the impact sound insulation performance of the floor slab can be greatly improved. FRP materials have the advantages of high strength, lightweight, and good corrosion resistance. They are more and more widely used in construction engineering. At this stage, for environmental friendly green building materials and nano-inorganic composite materials with certain effects, their main practice and application play an important role. It is proved that adding FBP material can greatly improve the impact sound insulation performance of floor slabs.

## 1. Introduction

Strengthening the overall cost management of green buildings can prevent serious waste of resources in engineering construction. At the same time, the standardized control of each link is realized while ensuring the quality and efficiency of project construction and reasonably controlling its construction period. In engineering construction, the basic characteristics and actual requirements of engineering construction should be analyzed to develop a practical and feasible comprehensive cost management work plan, achieve effective control of construction costs, and guarantee the economic benefits of the enterprise [1, 2]. The concept of “green building” has rich connotations; its genes contain a long history of regional architecture or climate-responsive design ideas. The energy crisis of the 20th century made clear the basic demands of “energy saving.” Energy-saving buildings represented by passive solar design have become its main form, and with the idea of sustainable development, the ideal of ecological architecture, which pursues the principles of the natural system, further deepens its connection with nature, and with the impact of the built environment on the health of its users, issues such as the close relationship between architecture and the space it creates and the development of human civilization are constantly being revealed. Human health, the inheritance of a human civilization, and natural “health” have been unified into the concept of “green building” [3]. Today, “green building” has become a composite concept that integrates multifaceted issues such as nature, culture, and the economy. Regarding the definition of green building, due to the differences in the economic development level, geographical location, and per capita resources of various countries, the international understanding of the definition and connotation of green building is not the same. The British Construction Equipment Research and Information Association (BSRIA) pointed out that for a green building that is conducive to people's health, its construction and management should be based on the principles of efficient resource utilization and ecological benefits [4].

The article "Impact Sound Insulation Performance Testing of Nano-Inorganic Composite Floor Slabs for Green Buildings" was retracted in 2023. Reasons: signs of a paper mill; suspected computer-generated content; unreliable results or conclusions; concerns about the data.

The indoor environment of civil buildings is often disturbed by various noises, among them, the interference from the upper floor slab, in particular, the interference of floor impact sound is widespread in many buildings, especially in residential buildings. The “Code for Design of Sound Insulation for Civil Buildings: GB 50118-2010” specifies detailed regulations on the impact sound insulation performance of floor slabs in six types of buildings, including residential buildings, schools, hospitals, hotels, offices, and commercial buildings. Taking residential buildings as an example, the weighted standardized impact sound pressure level of ordinary residential floor slabs should not exceed 75 dB, and those in high-requirement residential buildings should not exceed 65 dB [5]. At present, 100∼150 mm floor slabs of rough or dry-laid floor tiles cannot meet the impact sound insulation performance of floor slabs. The use of floating floor slabs can improve the impact sound insulation performance of floor slabs to a certain extent, but there are some defects, such as occupying effective storey height, increasing structural load, multiple construction steps, and high incremental cost. In recent years, Walshe K has conducted research on the sound insulation performance of sound insulation floating floor slabs [6]. Dong D. W. compared the performance of solid wood flooring, 20 mm thick XPS insulation board, and sound insulation floating floor slab [7]. For 5 mm sound insulation pad, 30 mm sound insulation mortar, and 30 mm thick composite foamed cement board, the performance of the five construction methods of 20 mm thick XPS insulation board and 5 mm thick sound insulation coating is compared by Homb A [8, 9]. An FRP (Fiber Reinforced Polymer, FRP) material is proposed, which has the advantages of high strength, lightweight, and good corrosion resistance. It is becoming more and more widely used in construction engineering. Experimental results show that with floor slabs using nano-inorganic composite material FBP, the impact sound insulation performance of the floor slab can be greatly improved. At this stage, for environmentally friendly green building materials and nano-inorganic composite materials with certain effects, their main practice and application play an important role.

The article "Impact Sound Insulation Performance Testing of Nano-Inorganic Composite Floor Slabs for Green Buildings" was retracted in 2023. Reasons: signs of a paper mill; suspected computer-generated content; unreliable results or conclusions; concerns about the data.

### 1.1. FRP Nano-Inorganic Composite Material Characteristics

FRP nano-inorganic composite material is made of multiple continuous fibers. There are three common types of FRP nano-inorganic composite materials: glass fiber, carbon fiber, and alamed fiber. Their chemical compositions are different.  Table 1 shows several performance parameters commonly used in the field of construction engineering [10].

As can be seen in Table 1, the density of these three FRP nano-inorganic composite materials is relatively small. This means that compared to steel, parts made of FRP nano-inorganic composite materials are lighter.

## 2. Application of FRP Nano-Inorganic Composite Materials in Construction Engineering

### 2.1. Protection System

Different forms of nano-inorganic composite materials have certain efficiency in their main practical applications and related target applications. The related protection system of nano-inorganic composite materials is feasible; therefore, the content of the entire structure and the selection of FRP nano-inorganic composite materials need to be based on the relevant requirements of the actual project and chosen according to certain demand information in order to ensure the feasibility of the actual application effect of the entire project. In addition, the entire project implementation and the application of nano-inorganic composite materials need to be carried out based on actual engineering requirements in order to meet the relevant requirements [11].

### 2.2. Decorative Structure

The FRP nano-inorganic composite materials can be made into different colors according to actual needs, of which the light transmittance is good. The processing factory can choose the appropriate color according to the overall tone of the actual placement position. After improving the processing technology and raw materials, the manufactured product can achieve 50% light transmittance. At the same time, FRP composite materials are closer to daily life and will not pollute nature. Compared with metal materials such as steel, which reduce the feeling of abnormal distance caused by metal, nano-inorganic composite materials will not pollute the environment during production, processing, and construction. The raw material of FRP material contains polymer, as a result, the entire material is difficult to degrade. Without deliberate damage, the application in landscape construction can significantly reduce the cost of manual maintenance, if damage occurs, repair and recovery are also very convenient. Therefore, FRP nano-inorganic composite materials have been widely used in urban landscape construction projects. In the environment of cold regions, the use of FRP decorative materials can also effectively resist the erosion of the building by the salt in the air and ice and snow, reduce maintenance costs, and extend the service life of the building [12].

The article "Impact Sound Insulation Performance Testing of Nano-Inorganic Composite Floor Slabs for Green Buildings" was retracted in 2023. Reasons: signs of a paper mill; suspected computer-generated content; unreliable results or conclusions; concerns about the data.

## 3. The Principle of the Sound Insulation Performance Test of the Impact Sound of the Floor Slab

At present, there are many kinds of methods for testing the sound insulation performance of floor slabs in China. This research uses a 1/3 octave band. the testing equipment is produced by Aihua Company, a professional acoustic testing manufacturer [13].

### 3.1. Test Principle

The on-site floor slab impact sound insulation performance test parameter is the standardized impact sound pressure level *L*_*nT*_′, *L*_*nT*_′ is the impact sound pressure level *L*_*i*_, subtract the correction term. The correction term is equal to the logarithm of the ratio between the reverberation time *T* and the reference reverberation time *T*_0_, measured in the receiving room, multiplied by 10, the unit is dB, and the calculation is shown in

(1) $$\begin{array}{c} L_{nT}=L_{i}-10\mathrm{lg}\frac{T}{T_{0}}, \end{array}$$

where *T* is the reverberation time measured in the receiving room. For house *T*_0_=0.5*s*. Taking the reference reverberation time 0.5 s for the standardized impact sound pressure level takes into account that the reverberation time of the residence is equal to 0.5 s.

It can be seen from the calculation formula of the above sound insulation, that if the weighted standardized impact sound pressure level *L*_*nT*_′ of a certain floor is tested, the measurement of the reverberation time *T* and the impact sound pressure level *L*_*i*_ of the measured floor room is the top priority. According to the test results of each parameter, substitute formula (1) for calculation, finally, the weighted standardized impact sound pressure level of the floor slab is obtained, and according to GBFF 50121-2005, carry out the classification of impact sound insulation performance. This research uses a 1/3-octave, fixed microphone test method. The test results of this detection method are more accurate and can be used as basic data for research [14].

The article "Impact Sound Insulation Performance Testing of Nano-Inorganic Composite Floor Slabs for Green Buildings" was retracted in 2023. Reasons: signs of a paper mill; suspected computer-generated content; unreliable results or conclusions; concerns about the data.

### 3.2. Test Method

#### 3.2.1. Measurement of Reverberation Time

Reverberation time is when the sound source starts to provide sound energy to the room, the time required for the sound pressure level to reach a steady state. In the field test of floor impact sound insulation performance, reverberation time needs to be tested . During the test, the doors and windows of the receiving room are required to be sealed, and the furniture is placed in place to simulate the real living environment and reduce the error of the test.

Reverberation time measurement in the receiving room: measuring the reverberation time of the receiving room requires at least 6 decay measurements for each frequency band. In each case, at least one loudspeaker position and three microphone positions should be used for two readings. According to IS0354 : 1985, the sound source stops sounding approximately at 0.1 s and then starts to calculate the reverberation time from the decay curve, or on the decay curve, the sound pressure level is calculated from a few decibels lower than the beginning of the decay. The decay range used must not be less than 20 dB and it should not be too large so that the observed decay cannot be close to a straight line. The lower end of the selected decay curve should be at least 10 dB higher than the background noise level [15].

#### 3.2.2. Test Method of Impactor and Microphone

*(1) Arrangement of the Equipment*. The impactors should be randomly distributed and placed at least 4 different positions on the floor to be tested. The distance between the position of the impactor and the boundary of the floor shall be ≥ 0.5 m.

*(2) Arrangement of Microphone*. The arrangement of microphones requires a distance of 0.7 m between the positions of the two microphones when arranging the microphones. The distance between any microphone and the room boundary or diffuser is 0.5 m, and the distance between any microphone and the test floor to be impacted is 1.0 m. Among them, fixed microphone positions: there should be at least 4 microphone positions, and they should be evenly distributed within the allowable range of the room to be tested.

*(3) Measure*. Fixed microphone measurement method: use a fixed microphone position to measure at least 6 times a combination of at least 4 microphone positions, and at least 4 impactor positions should be used. In the test, the author used 2 microphone positions and 2 impactor positions to form 4 possible combinations for measurement according to GB/T 19889.7-2005, the positions of the other two microphones and the two impactors are measured one-to-one.

## 4. Results and Analysis

When the floor surface material is selected as hard materials such as natural stone or ceramic floor tiles, the overall impact sound level of the floor slab is maintained at about 80 dB. The impact sound insulation performance of the floor slab is poor. It fails to meet the basic requirements of the design standard for impact sound insulation of green residential building floor slabs. This has become an urgent problem to be solved [16]. Through the test and analysis of the impact sound insulation performance of floor slabs with 4 methods in a certain area, specific results are as follows:

  ① In an ordinary residential area (furniture house), the floor slab method is leveling with 5 mm thick cement mortar + 120 mm thick reinforced concrete floor + 20 mm thick fine stone concrete is smoothed and polished. The on-site inspection result is the weighted standardized impact sound pressure level *L*_*nT*_′ of the floor slab. *w*=74  *dB*; the sound insulation performance is classified as level 2, and the test curve is shown in Figure 1 [17].
  ② In an ordinary residential area (mao embryo house), the floor plan is 30 mm thick fine-stone concrete + 20 mm-thick reinforced concrete floor + 20 mm thick concrete. The on-site inspection result is the weighted standardized impact sound pressure level *L*_*nT*_′ of the floor. *w*=73  *dB*; the sound insulation performance is classified as level 2, and the test curve is shown in Figure 2 [18].
  ③ In an ordinary residential district (fine decoration room), floor slab practice: 10 mm thick floor tiles + 4 mm thick construction glue cement mortar bonding layer + 40 mm thick C20 fine stone concrete + 20 mm thick nano-inorganic composite material FRP floor + 20 mm thick fine stone concrete with tamping and plastering + plaster ceiling. The on-site inspection result is the weighted standardized impact sound pressure level *L*_*nT*_′ of the floor. *w*=63  *dB*; the sound insulation performance is classified into 4 grades, and the test curve is shown in Figure 3.
  ④ In an ordinary residential area (adding carpets to the well-decorated rooms), floor practice: 20 mm thick carpet + 10 mm thick floor tiles + 4 thick construction glue cement mortar bonding layer + 40 mm thick C20 fine stone concrete + 20 mm thick nano-inorganic composite FRP floor + 20 mm thick fine stone concrete with tamping and smoothing + plaster ceiling. The on-site inspection result is the weighted standardized impact sound pressure level *L*_*nT*_′ of the floor. *w*=26  *dB*; the sound insulation performance is classified as 8 grades, and the test curve is shown in Figure 4.

The article "Impact Sound Insulation Performance Testing of Nano-Inorganic Composite Floor Slabs for Green Buildings" was retracted in 2023. Reasons: signs of a paper mill; suspected computer-generated content; unreliable results or conclusions; concerns about the data.

The above four types of floor slab practices are more common in rough or finely decorated residential buildings in a certain area. By comparing Figures 1 and 2, we found that the weighted standardized impact sound pressure level *L*_*nT*_′ of the reinforced concrete floor slab with the same thickness after adding the fine stone concrete floor slab. The increase of *w* is basically not large and can be ignored, therefore, it is necessary to take certain technical measures to improve the impact sound insulation performance of the floor slab in the rough room. By comparing Figures 3 and 4, in the currently popular finely decorated residences, by adding a common elastic material like carpet, the impact sound insulation performance of the floor slab can be greatly improved. This is due to the sound insulation effect of the elastic surface layer of the carpet (elastic floor) on the impact sound. The mass of the impact hammer and the elasticity of the flexible surface layer can be combined into a vibration system to consider, thus, the impact sound improvement value Δ*L* in the sound frequency range above the surface layer resonance frequency *f*_*R*_ is obtained. As

(2) $$\begin{array}{c} \Delta L=L_{N0}-L_{NR}=40\;\log\;{\text{fif}}_{R}\left(f>f_{R}\right), \end{array}$$

(3) $$\begin{array}{c} f_{R}=\frac{1}{2\pi \sqrt{M/D}}, \end{array}$$

where *L*_*N*0_ is impact sound pressure level of unpaved elastic surface floor slabs; *L*_*NR*_ is impact sound pressure level of laying elastic surface floor slab; *M* is the quality of the impact hammer; and *M*is the force (stiffness) required by the elastic surface unit to compress during the impact.

It can be seen from equation (2) that the improvement value of impact sound pressure level increases with the increase of frequency. The frequency is doubled and the improvement value is increased by 12 dB. Since the improvement value of high frequency in the elastic surface layer is very high, this kind of floor slab can be laid with an elastic surface layer such as carpet, which can greatly improve the sound insulation performance of its impact sound [19].

Looking at the trend of architectural development, its main development direction is to promote the safety and reliability of the building structure. At the same time, the building structure is more lightweight and beautiful. Therefore, fiber-reinforced nano-inorganic composite materials conform to this development trend, and they can meet the requirements of architectural development and design. According to the corresponding information, nano-inorganic composite materials have not been widely used in construction projects, mainly due to three aspects: (1) The manufacturing process of fiber-reinforced nano-inorganic composite materials is more complicated, as a result, their cost is very high and they are not suitable for large-scale applications and construction projects. (2) Due to the limitations of current science and technology, once the nano-inorganic composite material is scrapped, it cannot be used rationally. The high cost of recycling technology limits its wide application. (3) For the application process of nano-inorganic composite materials, because of the low-quality testing technology, they cannot be tested effectively. At present, there is a lack of systematic safety assessment methods for composite building structures and mature repair specifications for composite building structures. However, the development trend of nano-inorganic composite materials is gradually moving towards the direction of low cost and high technology [20].

The article "Impact Sound Insulation Performance Testing of Nano-Inorganic Composite Floor Slabs for Green Buildings" was retracted in 2023. Reasons: signs of a paper mill; suspected computer-generated content; unreliable results or conclusions; concerns about the data.

## 5. Conclusion

The rough state of the single-value evaluation of floor impact sound can reach ≤64 dB, and the finished state of floor tiles can reach ≤73 dB, meeting the specification requirements. When the delivery and acceptance of a few engineering projects require inspection on the surface of the sound insulation nano-inorganic composite material FRP, the designer proposes a reasonable standard weighted impact sound pressure level limit for the rough state. In order to ensure that the sound insulation performance after the decoration meets the standard requirements, a design margin of no less than 12 dB is required.

## Figures and Tables

**Figure 1:** The impact curve of the floor slab of an ordinary residential district (mao embryo house).

**Figure 2:** The catching curve of the floor slab of an ordinary residential district (mao embryo house).

**Figure 3:** Floor spreading curve of an ordinary residential community (finely decorated room).

**Figure 4:** The floor catching curve of an ordinary residential community (furnished room with additional carpet).

**Table 1:** FRP nano-inorganic composite material characteristics.

Type	Density	Elastic modulus	Tensile strength
Ordinary steel bar	7850	2.1*∗*106	400
Glass fiber	2000	5.1*∗*104	1670
Carbon fiber	1500	1.5*∗*106	1700
Alamed fiber	1300	6.4*∗*104	1610

## Data Availability

The data used to support the findings of this study are available from the corresponding author upon request.
